# Research on the Cultivation Path of Teenagers' Sports Health Literacy under the Background of Healthy China

This article has been retracted.

**DOI:** 10.1155/2022/3031475

**Published:** 2022-01-27

**Authors:** Yong Jiang, Guangjian Xu

**Affiliations:** ^1^Liaoning Normal University, Dalian, Liaoning Province 116028, China; ^2^University of Georgia, Athens, Georgia

## Abstract

Health literacy refers to an individual's ability to acquire and understand health information and use it to maintain and promote his own health. In physical education, teenagers' physical health literacy refers to teenagers improving their physical quality and comprehensive ability through physical training. The development of youth sports activities mainly depends on school physical education. Without the main channel of school physical education, it is difficult to achieve the strategic goal of improving youth health literacy. In order to effectively promote the cultivation of teenagers' health literacy, it is necessary to establish a scientific and reasonable physical education system according to the cultivation characteristics of teenagers' sports health literacy. Constantly strengthening the supervision of teenagers' physical exercise and paying attention to cultivating teenagers' sports habits are of great significance to the cultivation of teenagers' sports health literacy and their future study and development. Based on this, this paper expounds and analyzes the concept, necessity, and training path of teenagers' sports health literacy under the background of healthy China.

## 1. Introduction

In recent years, campus sports security incidents occur frequently, which has produced a certain shock and panic in the society. With the rapid development of social economy and the continuous improvement of people's living standards, on the premise that people's material conditions are met, health has become the main goal of people's pursuit, and health literacy has become an important indicator of social development [1]. Driven by the international situation, in order to improve the quality of their international talent training, countries have started to carry out core literacy research in different degrees and determined the content framework system of core literacy with different contents according to their own needs [2]. Health literacy refers to the ability of individuals to obtain and understand health information and use this information to maintain and promote their own health, and sports health literacy is an important part of health literacy [3]. In physical education teaching, teenagers' physical health literacy refers to teenagers' physical quality and comprehensive ability through physical training [4]. The development of national sports literacy is an important condition for teenagers' physical and mental health and the improvement of sports literacy level, and it is also an inevitable requirement for the great rejuvenation of the Chinese nation [5]. Youth sports health literacy is an important means to improve the level of physical health of young people. We need to fully combine the requirements of healthy China strategy and the connotation of sports health literacy and actively put forward effective training path to cultivate youth sports health literacy [6].

Under the background of healthy China strategy, we need to pay more attention to teenagers' health. As the future of the motherland and the hope of the nation, teenagers shoulder the important task of realizing healthy China and the Chinese dream. Therefore, it is very necessary to promote the cultivation of teenagers' sports health literacy [7]. It is not only an important way to strengthen the physical health of teenagers but also an important means to implement the healthy China strategy. The development of youth sports activity plan mainly depends on school sports. Without the main channel of school sports, it is difficult to achieve the strategic goal of improving youth health literacy [8]. The level of health literacy directly affects the speed and quality of people's all-round development and even affects the development of the whole society. Sports can not only strengthen the body but also play an important role in cultivating students' intelligence, aesthetic emotion, and strong will [9]. It is of great significance to continuously strengthen the supervision of teenagers' physical exercise and pay attention to the cultivation of teenagers' sports habits for the cultivation of teenagers' sports health literacy and their future learning and development [10]. This paper expounds and analyzes the concept, necessity, and training strategy of adolescent sports health literacy under the background of healthy China.

## 2. Connotation of Sports Health Literacy

Since the 21st century, sports events have become an important recreational activity and a topic of discussion after dinner. With the further spread of the influence of sports events, as educators, we should effectively combine sports events with sports culture and our own cultural literacy. It is proposed to strengthen physical education and extracurricular exercise to promote teenagers' physical and mental health and physical fitness. It can be seen that the development of students' physical quality has become a topic of concern to the whole society. At present, the annual test results of the Ministry of Education show that the physical quality of college students shows a downward trend. Starting from the sports events that students pay most attention to, we study the impact of sports events on students' sports cultural literacy, so as to improve students' sports knowledge, sports awareness, sports ability, and the development of sports personality.

At present, the low level of Chinese teenagers' sports health literacy is related to China's imperfect sports system. Therefore, in order to improve the health level of Chinese youth sports, we must improve the operation mechanism of youth sports. Sports literacy is a kind of sports quality formed by combining acquired social factors and sports ability on the basis of innate natural factors. It is divided into sports theory knowledge, sports appreciation and methods knowledge, and sports guidance knowledge. As an important means of health promotion, physical education should play an irreplaceable role in the realization of national health literacy goals. Health literacy refers to a kind of ability, the ability to use the health knowledge and skills to deal with health problems. The basis of examining whether a person has health literacy includes health concept, health behavior, health knowledge, and health skills. Sports health quality is an important reference index for citizens' health quality in a country. If a country's citizens' overall health quality is low, it will not only affect citizens' personal life and work but also have an impact on social and economic development. Health literacy is a comprehensive ability to maintain and promote health, and improving this comprehensive ability is the only way to promote health. Sports health knowledge is the basic condition for forming sports consciousness, while sports health consciousness is the main motive force for producing sports behavior, which is the important carrier of sports health consciousness and the result of sports health behavior.

The sports health literacy system composed of sports knowledge, sports consciousness, and sports behavior needs to be formed through different links and influencing factors. Sports health literacy includes sports health behavior, sports health knowledge, and sports health consciousness. Sports health behavior includes two important aspects: sports health civilized behavior and physical and mental exercise. Sports health knowledge includes fully understanding and mastering health views and concepts and effectively applying the basic knowledge of health in life, work, and study in different environments. Sports health consciousness mainly includes interest, values, views, aims, and emotions of sports. The promotion of health literacy can promote the improvement of adolescent health behavior, so as to effectively promote and manage adolescent health. Physical health is an important aspect of health, and the promotion of physical health is undoubtedly an important aspect of improving health literacy. The purpose of promoting adolescent physical health and improving health literacy is consistent and mutually based, and the means and ways are also interlinked. Sports literacy, as a high-level ideology, can be materialized as a kind of sports behavior, which improves the enthusiasm and enthusiasm of participating in physical exercise and plays an important role in improving teenagers' awareness, interest, and habit of physical exercise. The promotion of health literacy plays an important role in improving people's health management ability. It is necessary to guide teenagers to correctly understand health literacy and promote teenagers' health literacy and management.  Table 1 shows the sampling data analysis of students' physical health in a school in recent five years.

Teenagers' actual physical health literacy will not only have an important impact on the next generation but also affect the previous generation to a certain extent. In order to effectively play the connecting role of teenagers, it is necessary to pay attention to cultivating teenagers' physical health literacy. Although sports literacy research results have health literacy components, they tend to be sports content and lack of deep integration with health science. As far as sports health literacy is concerned, the formation process of individual sports health literacy is embedded in various sports events experienced in life, that is, sports experiences, and at the same time, individual sports health literacy is also shaped by these sports events. The core accomplishment of sports and health discipline is that students learn and master theoretical knowledge, sports skills, and sports and health methods by studying sports and health courses [12]. The core idea of management synergy theory, which emerged in the 1970s, is to deal with the correlation between elements so as to realize the unity of the whole system and improve the management efficiency. In a certain social environment, individuals have their own sports choices and sports health behaviors and can take advantage of their own sports health opportunities, overcome the constraints of social environment, and build and enhance their own sports health literacy. This is the connection between individual meaning and social meaning, and the coupling between individual needs and social needs.

## 3. The Cultivation Path of Teenagers' Sports Health Literacy under the Background of Healthy China

### 3.1. Pay Attention to the Cultivation of Teenagers' Physical Training Quality

In school education, it is necessary to make reasonable plans for school expenses and appropriately increase the funds for educational activities related to training teenagers' sports health literacy so as to create a good exercise environment and atmosphere for teenagers and encourage them to actively take physical exercise. Young people's sports health training is a systematic work, and any problems in any link will affect the realization of sports health training objectives. At present, China's sports health literacy mainly depends on school sports and interclass exercises, with sports classroom teaching as the mainstay, lacking of supervision mechanism and guarantee mechanism. Establishing the theoretical system of teenagers' sports health literacy is the basis of promoting teenagers' sports health literacy. When constructing the theoretical system of youth sports health literacy, we should take the knowledge of different fields and disciplines as the theoretical basis and combine with scientific analysis methods to enhance the scientific, rational, and feasible theoretical system.  Figure 1 shows the basic element structure of youth sports health literacy training system.

School is the place where teenagers come into contact with most frequently. In order to effectively cultivate teenagers' sports health literacy, it is necessary for schools to create a benign atmosphere of sports health education for teenagers at all levels, actively organize sports health lectures in schools, and invite professional sports health experts to popularize and educate teenagers' sports health knowledge. Compared with professional technology, physical education teachers' knowledge of health theory and education and teaching theory is weak. Schools should support teachers to participate in continuing education through various channels from the perspective of sustainable development and on the basis of encouraging individuals to learn by themselves. Schools create a good atmosphere for students to cultivate physical health, which can guide young people to acquire correct and professional health skills, so as to encourage young people to take more active physical exercise, and achieve self-strengthening through physical exercise, and gradually develop their own healthy lifestyle.

### 3.2. Create a Good Sports and Health Training Atmosphere for Young People

Under the background of healthy China, we should start with the life course factors that affect the youth's sports health literacy to improve the pertinence and effectiveness of the youth's sports health literacy cultivation. According to the characteristics and requirements of students, schools should improve the fun of physical education classes and enrich sports events. Secondly, according to the students' different goals at different stages, the corresponding teaching programs and teaching plans are formulated to improve students' enthusiasm for participating in sports. All aspects of the school should actively render the atmosphere of sports health education, and constantly invite university sports health experts to hold “sports health” lectures, and carry out popular science education knowledge transfer [13]. Through the implementation of sports health literacy training for young students, young people can know the correct sports health literacy knowledge, effectively judge the wrong sports health information to a certain extent, and reduce or avoid the risk factors that endanger physical and mental health in sports.  Figure 2 shows the relationship between the diversified cultivation of adolescent sports health literacy.

In the process of fully cultivating teenagers' sports health literacy, it is necessary to comprehensively monitor and scientifically evaluate the actual achievements of teenagers' sports health literacy. In order to scientifically evaluate teenagers' sports health literacy, it is necessary to establish an operable, flexible, and reliable monitoring and evaluation system to regularly monitor all aspects of teenagers' sports health literacy. In the process of realizing the combination of teenagers' physical fitness and health literacy, the integration of methods and models should be realized on the basis of theory to provide conditions for the constitution of teenagers' sports health literacy system.

## 4. Conclusions

The research on health literacy in China started relatively late and mostly concentrated on the research on health literacy of special groups and residents. Under the background of healthy China, in order to fully realize the cultivation of young people's sports health literacy, it is necessary to increase research on relevant groups, actively innovate more effective training paths, and comprehensively promote the effective implementation of the healthy China strategy by cultivating young people's sports health literacy. As the future of the motherland, teenagers' health determines the health status of the whole country in the future, is related to the rise and fall of the country and the nation, and plays an important role in practicing the strategy of healthy China. Under the background of healthy China, promoting teenagers' sports health literacy can not only improve teenagers' comprehensive quality and ability but also lay a foundation for their future study and growth. In the process of realizing the combination of teenagers' physical fitness and health literacy, the integration of methods and models should be realized on the basis of theory to provide conditions for the constitution of teenagers' sports health literacy system. Schools should constantly improve sports facilities, introduce some new sports, enrich teaching methods, apply modern information technology to sports teaching activities, break the previous single teaching mode, enrich teaching content, and improve the effectiveness of sports teaching.

## Figures and Tables

**Figure 1:** The basic element structure of the youth sports health literacy training system.

**Figure 2:** The relationship between the diversified cultivation of youth sports health literacy.

**Table 1:** Analysis of sampling data of students' physical fitness.

Particular year	Qualified		Good		Excellent	
	Number of people	Proportion (%)	Number of people	Proportion (%)	Number of people	Proportion (%)
2020	1591	81.9	232	11.9	120	6.2
2019	1615	85.7	248	13.2	21	1.1
2018	1577	79.6	379	19.1	24	1.2
2017	1632	82.1	324	16.3	31	1.6
2016	1599	83.9	281	14.8	25	1.3

## Data Availability

The data used to support the findings of this study are included within the article.

## References

[1] Rudolph C. W., Allan B., Clark M. (2021). Pandemics: implications for research and practice in industrial and organizational psychology. *Industrial and Organizational Psychology*.

[2] Fang Y., Dai Q. (2019). Student physical education classroom performance based on subject core literacy. Sports World. *Academic Edition*.

[3] Guo H. (2018). Discussion on the cultivation path of adolescent’s’ physical health under the background of healthy China. *Contemporary Sports Science and Technology*.

[4] Ojio Y., Mori R., Matsumoto K. (2021). Innovative approach to adolescent mental health in Japan: school‐based education about mental health literacy. *Early intervention in psychiatry*.

[5] Zheng L., Yao J. (2019). Research on the dilemma and path of student’s’ health literacy development under the background of healthy China strategy. *Journal of Electronic Engineering Institute*.

[6] Ge X., Liu Z. (2017). Analysis of risk factors related to health literacy and obesity of adolescents. *Chongqing Medical Journal*.

[7] Milona M., Janiszewska-Olszowska J., Szmidt M., Kłoda K., Olszowski T. (2021). Oral health related behaviors in relation to DMFT indexes of teenagers in an urban area of North-West Poland—dental caries is still a common problem. *International Journal of Environmental Research and Public Health*.

[8] He W., Han T. (2018). Research on adolescent sports health accomplishment from the perspective of life course. *Youth Sports*.

[9] Guo H. (2018). Research on the cultivation of physical education students’ health literacy under the background of healthy China. *Sports World (Academic Edition)*.

[10] Kafyra M., Kalafati I. P., Kumar S. (2021). Dietary patterns, blood pressure and the glycemic and lipidemic profile of two teenage, European populations. *Nutrients*.

[11] Chen M., Jeronen E., Wang A. (2021). Toward environmental sustainability, health, and equity: how the psychological characteristics of college students are reflected in understanding sustainable development goals. *International Journal of Environmental Research and Public Health*.

[12] Yang Q., Yuan X. (2019). International experience and enlightenment of health education curriculum reform in primary and secondary schools based on health literacy. *Journal of Physical Education*.

[13] Wang D., Li W., Lin L. (2019). Analysis of the impact of physical fitness services on improving public health literacy. *Western Leather*.

